The article "Ultrasonic Characteristics of Diastasis Recti Abdominis in Early Postpartum" was retracted in 2023. Reasons: suspected computer-generated content; unreliable results or conclusions; lack of ethics approval or compliance; missing or withdrawn patient consent.

# Ultrasonic Characteristics of Diastasis Recti Abdominis in Early Postpartum

**DOI:** 10.1155/2022/3273911

**Published:** 2022-02-22

**Authors:** Lina Tan, Suzhen Ran, Hongmei Dong, Jun Wei, Haitao Ran

**Affiliations:** ^1^Institute of Ultrasound Imaging, Chongqing Medical University, Chongqing 400010, China; ^2^Department of Ultrasound, Chongqing Health Center for Women and Children, Chongqing 401147, China; ^3^Chongqing Key Laboratory of Ultrasound Molecular Imaging, Chongqing 400010, China; ^4^Department of Ultrasound, The Second Affiliated Hospital of Chongqing Medical University, Chongqing 400010, China

## Abstract

**Objective:**

Explore the ultrasound characteristics of early postpartum Diastasis Recti Abdominis (DRA) and provide effective data support for its clinical diagnosis and treatment.

**Method:**

A total of 458 parturients who were diagnosed with DRA in the Chongqing Maternal and Child Health Hospital from December 2017 to September 2020 underwent postpartum ultrasound examinations. All of which were located at four points: 6 cm above the umbilicus (point 1), 3 cm above the umbilicus (point 2), umbilicus (point 3), and 3 cm below the umbilicus (point 4) to detect the interrectus distance (IRD) in the resting and sit-up state of the parturients postpartum and to study the differences in maternal age, weight, and ultrasound diagnosis of IRD at different stages after delivery.

**Results:**

The IRD values of the four measurement points in the resting state of the parturient were significantly greater than the IRD values in the sit-up state. And in the resting state, the IRD value (4.31 ± 1.07 cm) of the point 3 region was the largest, and there were significant differences at different stages of the postpartum women. At the same time, the IRD values of points 3 and 4 have significant differences in parturient of different ages. In addition, the IRD values of the four measurement points of overweight women were higher than those of nonoverweight women.

**Conclusion:**

The umbilicus is the best ultrasound evaluation point for early postpartum DRA. The IRD value at this point in the resting state can be used as reference data for evaluating early postpartum DRA, which provides a useful reference for rapid postpartum recovery of parturients.

## 1. Introduction

The human rectus abdominis muscle is an important muscle of the anterior abdominal wall. It protects the abdominal organs, maintains intra-abdominal pressure, participates in the completion of defecation, childbirth, vomiting, coughing, and other physiological functions, and can lower the ribs to help exhale. It can also cause functions such as forward flexion, lateral flexion, and spine rotation [1]. Diastasis recti abdominis (DRA) is a traumatic disease characterized by the separation of two rectus abdominis along the linea alba of the abdomen [2], mainly the sequelae of pregnancy [3].

During pregnancy, due to changes in hormone levels in the body, changes in the elasticity of tissue structure, and the enlarged uterus during pregnancy, the abdominal wall dilates and extends, and the rectus abdominis on both sides will separate from the position of the midline of the ventral midline (linea alba) to both sides. DRA during pregnancy is a common phenomenon. The latest research shows that the incidence of postpartum DRA in women of childbearing age in China is higher, which is 45.14% [4]. This brings a series of problems to women's physical and mental health, such as physical changes, lower back pain, pelvic floor dysfunction, and psychological stress. It can cause abdominal wall hernias that require surgical treatment in severe cases [5]. In recent years, with the advancement of society, the improvement of living standards, and the vigorous development of the field of postpartum rehabilitation medicine, a majority of physicians and patients have paid more and more attention to DRA.

At present, domestic and foreign studies [6–9] have proved that high-frequency ultrasound has a high resolution for muscle observation, and it is feasible and effective to observe morphological muscle changes with high-frequency ultrasound. The internationally recommended DRA objective detection method is ultrasound [10], the gold standard for diagnosing pregnancy DRA. The most common detection location is around the umbilical cord. This method can detect about 60% of cases [11], which is more objective, repeatable, and highly sensitive than traditional clinical examination.

However, there is no uniform diagnostic standard for DRA, and there is a lack of diagnosis and treatment standards for DRA. This study uses high-frequency ultrasound technology to measure and study the distance between multipoint spacing of rectus abdominis separation in the early postpartum period, analyze its characteristics and find the best measurement points, aiming to efficiently evaluate postpartum DRA through ultrasound, and provide an effective reference for standardized diagnosis and treatment of DRA.

## 2. Materials and Methods

### 2.1. Research Subjects

A total of 458 parturients who were clinically examined as DRA in Chongqing Maternity and Child Health Care Hospital from December 2017 to September 2020 (when measured by palpation in the supine position, the width of rectus abdominis interval was more than 2 fingers is the clinical criteria for the diagnosis of DRA [2]) and confirmed as DRA by ultrasound examination (rectus abdominis interval of more than 2.0 cm indicates diastasis rectus abdominis [12]) were collected. Informed consent was obtained from all patients, and this study was approved by the Institutional Review Boards (IRB) of Chongqing Medical University.

Inclusion criteria were as follows: (1) women of childbearing age 22 years and older; (2) primiparous women with no previous reproductive history, (3) no complications such as pregnancy-induced hypertension and gestational diabetes, and (4) examination time ≥ 6 weeks postpartum.

Exclusion criteria were as follows: (1) history of abdominal surgery; (2) History of abdominal wall hernia, gestational diabetes mellitus, and other diseases; (3) History of DRA diagnosis; and (4) abdomen fat too thick to cooperate with manual testing.

### 2.2. Ultrasonic Testing

PHILIPS EPIQ5 color Doppler ultrasound diagnostic apparatus was used; the linear array probe frequency was 5-12 MHz. 3.5-5 MHz convex array probe can be selected according to need and cooperate with wide-view imaging if necessary. Rath metrology standard was referenced, but measurement modifications were performed. The examinee takes the resting supine state and the initial sit-up state (that is, the knee is bent about 90°, and the head is lifted about 30° with both hands) for direct rectus abdominis scanning. The interrectus distance (IRD) [13, 14] was measured at four points: 6 cm above the umbilicus (point 1), 3 cm above the umbilicus (point 2), umbilicus (the lower edge of the probe is flat with the upper edge of the umbilicus when transected, point 3), and 3 cm below the umbilicus (point 4). Each measurement was repeated three times, the average value was taken as the final measurement value, and the data format is reserved to two decimal places, in centimeters (cm).

### 2.3. Statistical Analysis

Statistical analysis was performed using SPSS 22.0 software. Measurement data in accordance with normal distribution were expressed as mean ± standard deviation (SD), the *t*-test was used for comparison between two groups, and analysis of variance was used for multiple group comparison. Enumeration data were expressed by frequency (*n*) and percentage (%). *P* < 0.05 indicated a significant difference.

## 3. Results

### 3.1. Basic Patient Information

Four hundred and fifty-eight parturients were included, of whom 147 (32.1%) were 22-30 years old, 239 (52.18%) were 30-35 years old, and 72 (15.72%) were 35-42 years old. Postpartum examination time was between 6 and 8 weeks in 350 (76.42%), and 108 (23.58%) were more than 8 weeks. There were 167 persons (36.46%) with a BMI greater than or equal to 24 and 291 persons (63.54%) with a BMI less than 24 (Table 1).

### 3.2. Comparison of the IRD Values between the Resting State and the Sit-Up State of the Parturient

First, ultrasound was used to detect the IRD values of the parturient in different states. The results showed that the IRD values of the 4 measurement points of the parturient in the resting state were significantly greater than the sit-up state, and the IRD value measured at point 3 (4.31 ± 1.07 cm) was the largest (Table 2). In the sit-up state, the separation distance will be reduced with the contraction of the rectus abdominis.  Figure 1 shows the schematic diagram of ultrasound examination of the parturient positioned at different measurement points in the resting and sit-up state.

### 3.3. Comparison of IRD Values of Parturients at Different Stages

Further, the IRD values of the parturients of different ages, weights, and postpartum stages were compared under the resting state. The results show that in the resting state, the IRD values of points 3 and 4 were significantly different between different age groups, and the IRD values of each point tended to increase with age groups (Figure 2(a)). At the same time, the IRD value of each point showed a downward trend with the passage of postpartum time. And the IRD value of point 3 was significantly higher than that of 8 weeks in the 6-8 weeks postpartum group, but there was no significant difference in other localization areas (Figure 2(b)). In addition, the IRD values of the four measurement points in the BMI ≥ 24 kg/m^2^ group were higher than those of the parturients in the BMI < 24 kg/m^2^ group (Figure 2(c)).

## 4. Discussion

In recent years, ultrasound has been recognized as the gold standard for the non-invasive assessment of DRA [15]. IRD directly reflects the DRA, and the larger the distance, the more severe the degree of DRA [16]. Based on this, 458 postpartum women with DRA were included in this study, and the severity of DRA in the early postpartum period was determined by comparing the IRD values at different measurement points at rest and at different stages (age, weight, and time after delivery) by ultrasound scanning.

In the present study, we measured the IRD values of primiparous women at rest and sit-up state. It was found that the IRD was greatest at the umbilicus compared with other measurement points (3 cm above the umbilicus, 6 cm above the umbilicus, and 3 cm below the umbilicus) in the resting state. That is, it best reflects the severity of DRA objectively. Studies have shown that only 11% of DRA occurs below the umbilicus, while 52% of DRA is found at the umbilicus, and only 37% above the umbilicus, indicating the advantages of umbilical positioning [17]. Moreover, the umbilicus is the obvious anatomical landmark of the human body, which is the easiest to locate and has the least measurement error. The latest research also pointed out that the umbilical level IRD of the pelvic floor dysfunction (PFD) group was significantly greater than that of the non-PFD group. There was no statistically significant difference in the IRD of 3 cm above the umbilicus and 3 cm below the umbilicus between the two groups, suggesting obstetric factors (pregnancy and childbirth) has a more significant impact on the rectus abdominis at the umbilical level. DRA, especially at the umbilical level, affects the support function of the pelvic floor muscles and may promote the occurrence of PFD [18].

At the same time, this study conducted a comparative analysis of the IRD values in different age groups at the resting state and found that there was an increasing trend in IRD values with increasing age at all measurement points. However, the difference of this rising trend was statistically significant only at two measurement points, umbilical and 3 cm below the umbilicus. In addition, in the resting state, the IRD value of the overweight group (BMI ≥ 24 kg/m^2^) was significantly higher than that of the nonoverweight group (BMI < 24 kg/m^2^). The degree of DRA in the umbilical was the heaviest in the overweight group. Studies have shown that maternal age and weight gain are risk factors for DRA [19], which was consistent with the results of present study results.

The results of this study also indicate that the degree of DRA decreases with time after delivery. However, in the resting state, IRD values in the umbilicus only were significantly lower in the late postpartum period (i.e., >8 weeks) than in the early period (6-8 weeks). Studies have also shown that IRD decreased significantly at 8 weeks postpartum and plateaued [13]. The prevalence of DRA gradually decreased from 100% at 35 weeks of gestation to 52.4% at 6 weeks postpartum and 39.3% at 6 months postpartum, and there was also a gradual decrease in IRD at this stage [20]. This indicated a more severe degree of umbilical DRA in the early postpartum period.

However, this study still has certain limitations: (1) although the total sample size is large, it is a single-center study. (2) This issue of whether the intrinsic reason why the umbilicus becomes the most severe point for the occurrence of postpartum DRA compared with other measurement points is related to human posture, hormone secretion, pelvic floor structure, and mode of delivery needs to be confirmed by further studies.

## 5. Conclusion

In summary, the measurement of the anterior layer distance of the transumbilical rectus abdominis sheath in the resting state can be used as an efficient ultrasonic detection method for early postpartum DRA, which can reasonably evaluate the severity of DRA in the early postpartum period and provide some reference for standardized diagnosis and treatment of DRA.

## Figures and Tables

**Figure 1:** Schematic diagram of interrectus distance (IRD) ultrasound measurement at different measurement points. Point 1, 6 cm above the umbilicus; point 2, 3 cm above the umbilicus; point 3, umbilicus; and point 4, 3 cm below the umbilicus.

**Figure 2:** Comparison of interrectus distance (IRD) measurements of parturients at different stages in the resting state. (a) Comparison of IRD measurement values of maternal status 1 in different age groups, ^∗^*P* < 0.05, ^∗∗^*P* < 0.01 vs. 22-30 years old group. (b) Comparison of IRD measurement values of maternal status 1 at different postpartum examination times, ^∗^*P* < 0.05 vs. 6-8 weeks group. (c) Comparison of IRD measurement values of maternal status 1 in different BMI groups, ^∗∗^*P* < 0.01 vs. <24 group.

**Table 1:** Basic information of patients (*n* = 458).

Variables		Number of people	Percentage (%)
Age	22-30 years (not including 30 yr)	147	32.10
	30-35 years	239	52.18
	35-42 years (not including 35 yr)	72	15.72
Postpartum examination Examination time	6-8 weeks	350	76.42
	>8 weeks	108	23.58
BMI value	<24 kg/m^2^	291	63.54
	≥24 kg/m^2^	167	36.46

**Table 2:** Comparison of IRD values of two states at different measuring points.

Measuring point	Resting state (cm)	Sit-up state (cm)	*t* value	*P* value
Point 1	2.59 ± 0.99	2.10 ± 0.85	22.579	≤0.001
Point 2	3.48 ± 1.05	2.68 ± 0.84	26.354	≤0.001
Point 3	4.31 ± 1.07	2.99 ± 0.92	34.770	≤0.001
Point 4	2.51 ± 1.26	1.62 ± 0.96	24.378	≤0.001

Data are present as mean ± SD. Point 1, 6 cm above the umbilicus; point 2, 3 cm above the umbilicus; point 3, umbilicus; and point 4, 3 cm below the umbilicus.

## Data Availability

The data used to support the findings of this study are available from the corresponding author upon request.

## References

[1] Bai S. L. (2009). *Systematic Anatomy*.

[2] Michalska A., Rokita W., Wolder D., Pogorzelska J., Kaczmarczyk K. (2018). Diastasis recti abdominis - a review of treatment methods. *Ginekologia Polska*.

[3] Cardaillac C., Vieillefosse S., Oppenheimer A., Joueidi Y., Thubert T., Deffieux X. (2020). Diastasis of the rectus abdominis muscles in postpartum: concordance of patient and clinician evaluations, prevalence, associated pelvic floor symptoms and quality of life. *European Journal of Obstetrics, Gynecology, and Reproductive Biology*.

[4] Liu Y. L., Zhao Q. R., Li J. (2020). Incidence of postpartum diatasis recti abdominis in Chinese childbearing women-a meta analysis. *Chinese Journal of Public Health*.

[5] Sperstad J. B., Tennfjord M. K., Hilde G., Ellström-Engh M., Bø K. (2016). Diastasis recti abdominis during pregnancy and 12 months after childbirth: prevalence, risk factors and report of lumbopelvic pain. *British Journal of Sports Medicine*.

[6] Liu C. L., Zhang Z. J., Yu J. (2014). The reliability of abdominal muscle thickness measurement by rehabilitative ultrasound imaging in healthy youth. *Chinese Journal of Rehabilitation Medicine*.

[7] Tahan N., Khademi-Kalantari K., Mohseni-Bandpei M. A., Mikaili S., Baghban A. A., Jaberzadeh S. (2016). Measurement of superficial and deep abdominal muscle thickness: an ultrasonography study. *Journal of Physiological Anthropology*.

[8] Bentman S., O'Sullivan C., Stokes M. (2010). Thickness of the middle trapezius muscle measured by rehabilitative ultrasound imaging: description of the technique and reliability study. *Clinical Physiology and Functional Imaging*.

[9] Weis C. A., Triano J. J., Barrett J., Campbell M. D., Croy M., Roeder J. (2015). Ultrasound assessment of abdominal muscle thickness in postpartum vs nulliparous women. *Journal of Manipulative and Physiological Therapeutics*.

[10] Rath A. M., Attali P., Dumas J. L., Goldlust D., Zhang J., Chevrel J. P. (1996). The abdominal linea alba: an anatomo-radiologic and biomechanical study. *Surgical and Radiologic Anatomy*.

[11] Kimmich N., Haslinger C., Kreft M., Zimmermann R. (2015). Rektusdiastase und Schwangerschaft. *Praxis*.

[12] Wang Q., Yu X. J., Yang X. (2019). Risk factors for diastasis recti abdominis after delivery. *Progress in Obstetrics and Gynecology*.

[13] Coldron Y., Stokes M. J., Newham D. J., Cook K. (2008). Postpartum characteristics of rectus abdominis on ultrasound imaging. *Manual Therapy*.

[14] Pascoal A. G., Dionisio S., Cordeiro F., Mota P. (2014). Inter-rectus distance in postpartum women can be reduced by isometric contraction of the abdominal muscles: a preliminary case-control study. *Physiotherapy*.

[15] Keshwani N., Hills N., McLean L. (2016). Inter-rectus distance measurement using ultrasound imaging: does the rater matter?. *Physiotherapy Canada*.

[16] Theodorsen N. M., Strand L. I., Bø K. (2019). Effect of pelvic floor and transversus abdominis muscle contraction on inter-rectus distance in postpartum women: a cross-sectional experimental study. *Physiotherapy*.

[17] Thabet A. A., Alshehri M. A. (2019). Efficacy of deep core stability exercise program in postpartum women with diastasis recti abdominis: a randomised controlled trial. *Journal of Musculoskeletal & Neuronal Interactions*.

[18] Wang J., Wang X., Gu J. J., Li H. (2020). Ultrasond examination in evaluation of structure and function of rectus abdominis and pelvic floor in early postpartum women. *Chinese Journal of Interventional Imaging and Therapy*.

[19] Gitta S., Magyar Z., Tardi P. (2017). Prevalence, potential risk factors and sequelae of diastasis recti abdominis. *Orvosi Hetilap*.

[20] Fernandes da Mota P. G., Pascoal A. G., Carita A. I., Bø K. (2015). Prevalence and risk factors of diastasis recti abdominis from late pregnancy to 6 months postpartum, and relationship with lumbo-pelvic pain. *Manual Therapy*.

